# Unilateral Biportal Endoscopic Discectomy versus Microendoscopic Discectomy for the Treatment of Lumbar Spinal Stenosis: A Systematic Review and Meta-Analysis

**DOI:** 10.1155/2022/7667463

**Published:** 2022-09-21

**Authors:** Yufei Niu, Zhen Shen, Haoyang Li

**Affiliations:** Department of Orthopaedics, Jincheng people's Hospital, Jincheng, China

## Abstract

**Objective:**

In minimally invasive spinal surgery, the treatment of lumbar spinal stenosis with microendoscopic discectomy (MED) or unilateral biportal endoscopic discectomy (UBED) shows effective results, but which is more effective is controversial. Our study aimed to evaluate the efficacy and safety of UBED versus MED in the treatment of lumbar spinal stenosis by a systematic review and meta-analysis, so as to provide reference for the promotion of UBED in clinical practice.

**Methods:**

The multiple databases like PubMed, EMBASE, Web of Science, Cochrane Library, Chinese National Knowledge Databases, Chinese BioMedical Database, and Wanfang Database were used to search for the relevant studies. Review Manager 5.4 was adopted to estimate the effects of the results among selected articles. Odds ratio (OR) and mean difference (MD) with 95% confidence intervals (CIs) were used to estimate the overall pooled effect. Subgroup analysis, forest plots, funnel plots and Egger's test for the articles included were also conducted.

**Results:**

Three randomized clinical trials and seven cohort studies were finally retrieved, these studies included 685 and 829 patients in the UBED and MED groups, respectively. There were no differences in terms of operation time (MD = -0.92, P =0.72), estimated blood loss (MD = -26.31, P =0.08), complications (MD =0.81, P =0.38) and Oswestry Disability Index (ODI) score (P >0.05 in four subgroup) between the two groups. The visual analog scale (VAS) score of back pain in the UBED group was better than MED group only at 6 months (MD = -0.23, P =0.006) after operation, the VAS score of leg pain in the UBED group was better than that of MED group at 3 mouths (MD = -0.22, P =0.002) and 6 months (MD = -0.24, P =0.006) after operation, the UBED group had a less postoperative length of stay than the MED group (MD = -1.85, P <0.001). The bias analysis showed that there was no potential publication bias in the included literature.

**Conclusion:**

This study showed that compared with MED, UBED has the advantages of short hospital stay and good short-term curative effect, but there is no significant difference in long-term efficacy and safety, they can be replaced by each other in clinical application.

## 1. Introduction

Lumbar spinal stenosis is a common disease in spinal surgery, which tends to occur in middle-aged and elderly patients over 50 years old [1]. With the increase of age, the incidence rate also increases. It is considered to be the second largest cause of low back and leg pain in middle-aged and elderly people [2, 3]. Lumbar spinal stenosis refers to the changes in the morphology and tissue structure of lumbar bones and soft tissues (vertebral body, facet joint, lamina etc.) caused by various reasons, it usually results in stenosis of central spinal canal and lateral recess, causes nerve root and or cauda equina nerve to be stimulated or compressed, and results in clinical symptoms such as lower limb radiative pain and intermittent claudication, which seriously affects the quality of life of patients [4].

Traditional open laminectomy has a definite effect, but the operation extensively destroys the soft tissue structure, which will lead to long-term back heaviness and soreness, even some patients with poor physical conditions cannot tolerate spinal surgery [5]. At present, the clinical treatment of lumbar spinal stenosis is mainly single channel endoscopic surgery, including percutaneous foraminal endoscopic surgery and microendoscopic discectomy (MED) [6, 7]. These methods can completely preserve the physiological structure of the lumbar spine with small surgical trauma and fast postoperative recovery [8, 9]. However, there are also defects such as small scope of visual field under the microscope, limited operation under the microscope, and it is difficult to expand the range of decompression when necessary [10, 11].

Unilateral biportal endoscopic discectomy (UBED) is a new minimally invasive surgery for the treatment of lumbar spinal stenosis in recent years [12]. In the past decade, UBED has received the attention of clinicians under the improvement of Korean scholars [13–16]. This surgical method constructs two channels, one is implanted into the endoscope to provide vision, and the other is implanted into the surgical instrument operation, which combines the advantages of traditional minimally invasive surgery and open surgery [17].

Compared with conventional surgery for lumbar spinal stenosis, minimally invasive spinal surgery using microscope or endoscopic approach shows more effective clinical results [18, 19]. However, in minimally invasive spinal surgery, there has been a controversy about which is more effective in the treatment of lumbar spinal stenosis with microscope or endoscope [20, 21]. Through the systematic review and meta-analysis, this paper evaluated and compared the effect results of UBED versus MED in minimally invasive spinal surgery, and evaluated the effectiveness and safety of the two methods.

## 2. Methods

### 2.1. Literature Search Strategy

We searched the PubMed, EMBASE, Web of Science, Cochrane Library, Chinese National Knowledge Databases, Chinese BioMedical Database, and Wanfang Database, which were assessed up to June 2022 with the following keywords: (“unilateral biportal endoscopic discectomy” or “unilateral biportal endoscopic spinal surgery” or “unilateral biportal endoscopic laminectomy”) and (“microendoscopic discectomy” or “microscopic lumbar decompression laminectomy” or “micro endoscopic spine surgery”) and (“lumbar spinal stenosis”). There were no restrictions on the language of publication in document retrieval. We retrieved potentially relevant articles and screened their reference lists to find studies that our search strategy may have missed.

### 2.2. Study Selection

The potential relevant studies identified were retrieved and the respective full text analyzed for their eligibility according the PICOS criteria: (P) Population: patients with the lumbar spinal stenosis. (I) Intervention: patients underwent surgical corrections using the surgical approaches of unilateral biportal endoscopic discectomy (UBED). (C) Comparison: microendoscopic discectomy (MED). (O) Outcomes: intraoperative and postoperative indexes (operation time, estimated blood loss, postoperative length of stay, postoperative complication rate) and effectiveness indicators, such as the visual analog scale (VAS) score of back pain and leg pain, the Oswestry Disability Index (ODI) score. (S) Study design: clinical human studies, including randomized controlled trials (RCTs), retrospective cohort studies (RCSs), prospective cohort studies (PCSs) and case series.

### 2.3. Data Extraction and Quality Assessment

Two pairs of reviewers (Y Niu, Z Shen) independently screened titles, abstracts, and full-text articles of potentially eligible studies and resolved disagreement through discussion. The first author and the year of the study were extracted as general information. Parameters, such as country, study design, population number, gender, age, time of follow-up and study duration, were utilized to analyze the study characteristics.

The Newcastle Ottawa scale (NOS) and the Cochrane Collaboration's tool were used to evaluate the methodological quality and bias risk of non randomized controlled trials (nRCTs) and RCTs, respectively.

### 2.4. Statistical Analysis

Meta analysis was performed by using Review Manager 5.4 (Nordic Cochrane Centre). Briefly, we utilized the odds ratio (OR) with 95% confidence intervals (CIs) for dichotomous variables and mean difference (MD) with 95% CIs for continuous variables to estimate the overall pooled effect. We conducted the subgroup analysis according to the different follow-up time. The heterogeneity among trials evaluated by the *χ*^2^-based Q testing (0.05 was set as the statistical significance cut-off for the test of heterogeneity) and I^2^ statistics (I^2^>50%). In our analytical framework, fixed effect model or random-effect model was used depending on the absence (P >0.05 or I^2^<50%) or presence of significant heterogeneity. Funnel plot and Egger's test were used to show potential publication bias.

## 3. Results

### 3.1. Search Process

Figure 1 showed the process of screening articles for inclusion in the systematic review and meta-analysis. The search strategy resulted in a total of 820 articles from all databases. After duplicate elimination, 695 studies underwent titles and abstracts screening, leaving 96 articles for eligibility screening. After full-texts screening, 10 studies were finally included in our meta-analysis [22–31].

### 3.2. Characteristics of the Included Studies

The baseline characteristics of the patients included in the meta-analysis were reported in Table 1. This study included 3 RCTs [26, 29, 30], 5 RCSs [22, 23, 25, 27, 28] and 2 PCSs [24, 31], which included 685 patients treated with UBED and 829 patients treated with MED. The average age of each group was over 60. All the 10 articles were published from 2018 to 2021. The follow-up time were more than 6 months and the longest was more than 3 years.

### 3.3. Results of Quality Assessment

Finally, 3 RCTs and 7 cohort studies were included in this study. The Cochrane collaboration's tool and NOS were used to carry out the quality assessment. The results were shown in Tables 2 and 3, respectively. The quality of the three RCTs was high, and there were no obvious risk of bias. The final scores of the seven cohort studies were higher than 7 according to NOS, which represented that the bias of the 7 included literature was relatively small.

### 3.4. Primary Outcomes

#### 3.4.1. VAS (Back Pain)

Eight studies had data available to assess change in VAS of back pain. Although the overall combined effect showed that the VAS score (back pain) of UBED group was lower than that of MED group (MD = -0.36, 95% CI -0.66 to -0.05, P =0.02) (Figure 2), according to the different follow-up time, the VAS score (back pain) in UBED group was significantly lower than that of MED group at 6 months (MD = -0.24, 95% CI -0.40 to -0.07, P =0.006) after operation, but there was no difference between the two groups at 1 months (MD = -0.23, 95% CI -0.67 to 0.20, P =0.29), 3 months (MD = -0.48, 95% CI -1.03 to 0.08, P =0.09) and 1 year (MD = -0.31, 95% CI -1.01 to 0.39, P =0.38) after operation.

#### 3.4.2. VAS (Leg Pain)

For VAS of leg pain, 7 studies reported it. Meta-analysis showed that there was no significant difference of VAS score (leg pain) between UBED group and MED group (MD = -0.31, 95% CI -0.74 to 0.12, P =0.15) (Figure 3), however, after stratification according to the follow-up time, the subgroup meta-analysis showed that there was no significant difference of VAS score (leg pain) between the two group at 1 month (MD = -0.03, 95% CI -0.91 to 0.85, P =0.95) and 1 year (MD = -0.37, 95% CI -1.35 to 0.61, P =0.45) after operation, but the VAS score (leg pain) in UBED group was lower than that in Med group at 3 months (MD = -0.22, 95% CI -0.35 to -0.08, P =0.002) and 6 months (MD = -0.24, 95% CI -0.40 to -0.07, P =0.006) after operation.

#### 3.4.3. ODI

A total of 9 literature studies reported ODI. The overall combined effect showed that the ODI score of UBED group was lower than that of MED group (MD = -1.73, 95% CI -3.40 to -0.07, P =0.04) (Figure 4). However, according to the hierarchical comparison of different follow-up times, it was found that there was no significant difference in ODI value between the two groups in 1 month (MD = -3.62, 95% CI -8.18 to 0.93, P =0.12), 3 months (MD = -1.12, 95% CI -2.29 to 0.06, P =0.06), 6 months (MD = -0.72, 95% CI -0.19 to 1.63, P =0.12) and 1 year (MD = -2.59, 95% CI -6.92 to 1.75, P =0.24) after operation.

### 3.5. Secondary Outcomes

#### 3.5.1. Operation Time

Five studies comprising 1654 patients provided information regarding operative time. The UBED group showed no significant difference of operation time comparing to the MED group (MD = -0.92, 95% CI -5.97 to 4.13, P =0.72) (Figure 5).

#### 3.5.2. Postoperative Length of Stay

The postoperative length of stay was reported in 4 studies. The pooled data revealed that the postoperative length of stay was significantly shorter in the UBED group than the MED group (MD = -1.85, 95% CI -2.53 to -1.17, P <0.00001) (Figure 6).

#### 3.5.3. Estimated Blood Loss

For the estimated blood loss, 4 included studies reported it. The pooled result showed that the UBED group had no significant difference of estimated blood loss than the MED group (MD = -26.31, 95% CI -55.47 to 2.85, P =0.08) (Figure 7).

#### 3.5.4. Complication

The complication was reported in 6 studies. The pooled data revealed that no significant difference in the rate of complication was detected between the UBED group and the MED group (MD =0.81, 95% CI 0.51 to 1.29, P =0.38) (Figure 8).

### 3.6. Publication Bias

Funnel plot was performed to qualitatively evaluate the publication bias for the complication rate, The funnel plot seemed to be asymmetric (Figure 9), but the *P* value of Egger's test of quantitative analysis was >0.05, indicating that there was no obvious publication bias.

## 4. Discussion

The purpose of surgical treatment of lumbar spinal stenosis is to completely decompress the “responsible segment”, so that the compressed spinal cord and nerve roots can be effectively loosened, and at the same time, the overall stability of the spine can be destroyed as little as possible, so as to achieve the purpose of alleviating the symptoms of patients [32, 33]. Total laminectomy, which is commonly used in clinic, has the advantages of sufficient decompression, large operating space and clear vision, but it also has the disadvantages of large injury, long operation time and prone to lumbar instability or spondylolisthesis in the later stage [34]. Therefore, some patients need to perform spinal internal fixation and fusion at the same time, which prolongs the operation time and increases the cost of patients [35].

With the development of minimally invasive surgery, MED technology has gradually become a common method for the treatment of lumbar spinal stenosis [36]. It has the advantages of small incision, fast recovery, less bleeding, preservation of spinal soft tissue structure and so on [37]. However, the shortcomings of MED technology are also very obvious, such as the limited vision of surgery, and the limited range of motion of the instrument through a single channel. UBED combines the advantages of microscope and endoscope [38, 39]. UBED technology has two channels, one channel provides surgical field of vision and continuous flushing, and the other channel is used for instrument operation [40]. A separate operation channel increases the movable range of the operation, makes the operation easier, and also provides a good field of vision in the contralateral intervertebral foramen area [41, 42]. The continuous flushing function is conducive to controlling bleeding and providing a clearer surgical field of vision. UBED does not need a sleeve and will not restrict the use of instruments [43]. Conventional arthroscopic instruments and spinal open surgery instruments can be used, which can save costs [44].

In this study, the clinical outcome indicators of minimally invasive spinal surgery performed by UBED versus MED were combined analyzed, and a total of 10 literatures were included. In terms of effectiveness, compared with MED group, the VAS score (leg pain) of UBED group was better than MED group only at 3 and 6 months after operation, while there was no difference in other follow-up time between the two groups; at 6 months after operation, the VAS score (back pain) of UBED group was better than that of the MED group, while there was no difference in other follow-up time between the two groups. At any follow-up time, there was no significant difference in ODI between the two groups. Among the surgery related indicators, the postoperative length of stay in the UBED group was significantly lower than that in the MED group, but there was no difference in operation time, estimated blood loss and complication rate. Tang's research specifically made a meta-analysis of the postoperative complications of minimally invasive spinal surgery performed by UBED and MED [45]. The results showed that there was no statistical difference in the total complications between the two groups, which was consistent with our research results. Moreover, Chen's study also made a grouping analysis of the detailed complications, the results showed that there was no difference in the incidence of related complications such as epidural hematoma, nerve root injury, dural sac injury and incomplete decompression [46].

There were some limitations in this meta-analysis. Firstly, the included literature included 3 RCTs and 7 cohort studies. More observational studies were included in this study, which will limit the quality of the meta-analysis. Secondly, among the 10 literatures included, 7 were from South Korea, which may lead to certain limitations in the extrapolation of results. In addition, due to the small number of included literatures, this study did not make a detailed analysis of different types of complications, and some outcome variables were included in fewer literatures, which will also affect the reliability of the final conclusion.

## 5. Conclusions

To sum up, UBED has a faster recovery time than MED in the treatment of lumbar spinal stenosis, and the short-term (3 months and 6 months after operation) surgical effect is better, but the follow-up of 1 month and 12 months after operation shows that there is no significant difference, indicating that UBED and MED have the same curative effect in the treatment of lumbar spinal stenosis. However, due to the limitations of the quantity and quality of the included studies, the above conclusions still need to be confirmed by more high-quality studies.

## Figures and Tables

**Figure 1:** Schematic of the trial selection process.

**Figure 2:** Forest plots of patient clinical outcomes: VAS of back pain. VAS, visual analog scale. UBED, unilateral biportal endoscopic discectomy; MED, microendoscopic discectomy.

**Figure 3:** Forest plots of patient clinical outcomes: VAS of leg pain. VAS, visual analog scale. UBED, unilateral biportal endoscopic discectomy; MED, microendoscopic discectomy.

**Figure 4:** Forest plots of patient clinical outcomes: ODI. ODI, Oswestry Disability Index. UBED, unilateral biportal endoscopic discectomy; MED, microendoscopic discectomy.

**Figure 5:** Forest plots of patient clinical outcomes: operation time. UBED, unilateral biportal endoscopic discectomy; MED, microendoscopic discectomy.

**Figure 6:** Forest plots of patient clinical outcomes: postoperative length of stay. UBED, unilateral biportal endoscopic discectomy; MED, microendoscopic discectomy.

**Figure 7:** Forest plots of patient clinical outcomes: estimated blood loss.

**Figure 8:** Forest plots of patient clinical outcomes: complication. UBED, unilateral biportal endoscopic discectomy; MED, microendoscopic discectomy.

**Figure 9:** Funnel plot for potential publication bias of complication.

**Table 1:** Characteristics of included studies.

Study	Country	Study design	No. of patients		Gender (M/F)		Age (years)		Follow-up (months)	Duration
			UBED	MED	UBED	MED	UBED	MED		
Heo [24]	Korea	PCS	46	42	18/28	16/26	65.8 ± 8.9	63.6 ± 10.5	>12	March 2016 to October 2017
Choi [22]	Korea	RCS	35	30	14/21	17/13	65.4 ± 11.8	65.2 ± 12.0	6	December 2013 to March 2015
Heo [23]	Korea	RCS	37	33	15/22	12/21	66.7 ± 9.4	63.4 ± 11.1	12	March 2016 to December 2017
Kang [26]	Korea	RCT	32	30	18/14	14/16	65.1 ± 8.6	67.2 ± 9.5	6	January 2015 to December 2016
McGrath [28]	USA	RCS	50	45	27/23	27/18	—	—	12	September 2014 to February 2017
Park [30]	Korea	RCT	32	32	13/19	18/14	66.2 (41 – 80)	67.1 (45 – 79)	12	November 2017 to June 2018
Rieger [31]	Germany	PCS	327	413	152/101	178/119	76 ± 10	78 ± 13	12~36	January 2012 to July 2017
Kim [27]	Korea	RCS	30	30	13/17	12/18	64.23 ± 5.26	66.20 ± 6.01	12	September 2015 to March 2017
Min [29]	Korea	RCT	54	35	27/27	19/16	65.74 ± 10.52	66.74 ± 7.96	>36	March 2015
Ito [25]	Japan	RCS	42	139	28/14	71/68	66.3 ± 12.3	65.0 ± 11.1	>6	November 2018 to June 2019

UBED, unilateral biportal endoscopic discectomy; MED, microendoscopic discectomy; PCS, prospective cohort study; RCS, retrospective cohort study; RCT, randomized controlled trial.

**Table 2:** Risk of bias of randomized controlled trials.

Study	Random allocation	Hidden distribution	Blind method	Incomplete outcome data	Selective reporting of results	Other bias	Quality level
Kang [26]	Low risk	Low risk	Low risk	Low risk	Low risk	Low risk	High
Park [30]	Low risk	Low risk	Low risk	Low risk	Low risk	Low risk	High
Min [29]	Low risk	Low risk	Low risk	Low risk	Low risk	Low risk	High

**Table 3:** Risk of bias of cohort studies.

Study	Selection				Comparability of cohorts	Outcomes			Score^∗^
	Representativeness of cohort	Selection of nonexposed cohort	Ascertainment of exposure	Outcome lacking at the beginning		Outcome assessment	Sufficient follow-up time	Follow up adequacy	
Heo [24]	+	+	+	+	++	—	+	+	8
Choi [22]	+	+	+	+	++	+	+	+	9
Heo [23]	+	+	+	+	+	+	+	+	8
McGrath [28]	+	+	+	+	+	+	+	+	8
Rieger [31]	+	+	+	+	++	+	+	+	9
Kim [27]	+	+	+	+	+	—	+	+	7
Ito [25]	+	+	+	+	++	+	+	+	9

^∗^, The total score of NOS evaluation is 9 points; +, represents that the item has obtained the score; -, represents that the item has not been scored.

## Data Availability

The datasets used and analyzed during the current study are available from the corresponding author upon reasonable request.

## Abbreviations

MED: Microendoscopic discectomy
UBED: Unilateral biportal endoscopic discectomy
OR: Odds ratio
MD: Mean difference
CIs: Confidence intervals
ODI: Oswestry disability index
VAS: Visual analog scale
PICOS: Population, intervention, comparison, outcomes, study design
RCTs: Randomized controlled trials
RCSs: Retrospective cohort studies
PCSs: Prospective cohort studies
NOS: Newcastle Ottawa scale.
